The article "MUC1 gene silencing inhibits proliferation, invasion, and migration while promoting apoptosis of oral squamous cell carcinoma cells" was retracted in 2020. Reason: manipulated images.

# MUC1 gene silencing inhibits proliferation, invasion, and migration while promoting apoptosis of oral squamous cell carcinoma cells

**DOI:** 10.1042/BSR20182193

**Published:** 2019-09-16

**Authors:** Ai-Min Zhang, Xiao-Hui Chi, Zu-Qiang Bo, Xiao-Fang Huang, Jin Zhang

**Affiliations:** Department of Stomatology, Dongying City People’s Hospital, Dongying 257091, P.R. China

**Keywords:** Apoptosis, Invasion, Migration, MUC1 gene silencing, Oral squamous cell carcinoma, Proliferation

## Abstract

The aim of the present study is to investigate the role of RNA interference in the inhibition of MUC1 gene expression in occurrence and metastasis of oral squamous cell carcinoma (OSCC) and its in-depth mechanisms. The OSCC and normal oral mucosa tissues, as well as normal oral epithelial cell line HOK and OSCC cell line SCC-4, Cal-27, TSCCA, Tca8113 were obtained to detect the expression of MUC1. Slug expression in OSCC and normal oral mucosa tissues was also determined. The OSCC cells were grouped to investigate the role of MUC1 gene silencing on proliferation, DNA replication, cell cycle distribution, apoptosis, colony formation ability, epithelial-mesenchymal transition (EMT), invasion, and migration of OSCC cells. We first found higher positive rate of MUC1 and Slug expression in OSCC tissues. Next, it was determined that higher expression of MUC1 was found in OSCC tissues and cells. Furthermore, silencing of MUC1 declined Slug expression, inhibited the proliferation, DNA replication, cell cycle progression, and EMT while inducing apoptosis of OSCC cells. Our study suggests that overexpression of MUC1 is found in OSCC, and MUC1 gene silencing could inhibit the proliferation, invasion, and migration while inducing apoptosis of OSCC cells.

## Introduction

Oral squamous cell carcinoma (OSCC) is involved in the oral tongue, lower gingival and alveolus, upper gingival, floor of the mouth, retromolar triangle, buccal mucosa, lip mucosa, and hard palate [1]. OSCC accounts for nearly 3% of all malignant tumors around the world, with 550,000 new cases every year worldwide in recent years [2,3]. Smoking and alcohol consumption are regarded as the major risks for OSCC, but only a small part of people develop oral cancer with these habits, which suggests that other genetic factors also result in the pathogenesis of the disease [4,5]. Until now, the main therapy for OSCC is the surgical resection accompanied by radiotherapy and chemotherapy [6]. Great advances have been achieved in general patient care, surgical techniques, as well as local and systemic adjuvant therapies, while the mortality rate of OSCC still high and the 5-year overall survival rate remains less than 50% [7,8]. Based on this, it is of great importance to find potential targets for the treatment of patients suffering from OSCC [9].

The article "MUC1 gene silencing inhibits proliferation, invasion, and migration while promoting apoptosis of oral squamous cell carcinoma cells" was retracted in 2020. Reason: manipulated images.

Mucins, as high molecular weight glycoproteins, exert function in cell growth, differentiation and cell signaling, and the gene expression of mucin is highest in the system of respiratory, digestive, and reproductive systems [10–12]. Mucin 1 (MUC1) is a membrane-bound protein, and it is a member of the mucin family [13]. MUC1 possesses a core protein mass of 120–225 kDa, which increases to 250–500 kDa with glycosylation [14–16]. MUC1 consists of two subunits, namely an N-terminal extracellular subunit (MUC1-N) together with a C-terminal transmembrane subunit (MUC1-C) [17]. It is reported that overexpression of MUC1 is able to induce anchorage independent growth and tumorigenicity [18]. Meanwhile, an aberrant expression of MUC1 has highlighted its role in the pathogenesis of various human cancers [10]. Recent article has described that MUC1 might serve as a regulator engaging in several interactions that could contribute to enhance migration and invasion, as well as survival [19]. It is also reported that MUC1 is presented on the majority of cancers with glandular epithelial origin, which acts as a potential target for therapeutic interventions in these cancers [20]. A recent study has demonstrated that MUC1 expression might be a useful diagnostic target for prediction and treatment of the invasive/metastatic potential of OSCC [21]. Slug (Snail2) plays essential roles in controlling the epithelial-mesenchymal transition (EMT) during disease development [22]. Evidence has shown that MUC1 may up-regulate EMT-related genes such as Snail and Slug [23]. However, no study focussed on the silencing of MUC1 on the biological functions of OSCC cells. Based on this, we conducted the present study to investigate the role of RNA interference in the inhibition of MUC1 expression in occurrence and metastasis of OSCC.

## Materials and methods

### Study subjects

The samples were collected from 90 cases of OSCC who were surgically resected from the Dongying City People’s Hospital from 2016 to 2017. Case selection was based on availability organization and tracking data. Of these patients, 46 were males and 44 were females, aged 32–74 years, with an average age of 55.21 ± 0.29 years. Patients received no preoperative radiotherapy, chemotherapy, biotherapy, or other specific treatment for cancer. According to World Health Organization (WHO) pathological classification amongst those 90 OSCC patients, there were 30 cases of well differentiation, 30 cases of moderate differentiation, and 30 cases of poor differentiation. According to the TNM staging of the International Union Against Cancer (UICC) in 2009 [24], there were 60 cases in N0 phase, 27 cases in N1 phase, and three cases in N2 phase. The OSCC tissues were selected as an experimental group. Additionally, 35 cases of normal oral mucosa tissues (patients with traumatic or orthodontic extraction without smoking and drinking history) were used as a control group. All tumor cases were reassessed and histologically classified by the same pathologist. Histological identification was based on WHO standards. The Medical Ethics Survey Association of Dongying City People’s Hospital authorized the study and the patient informed consent was obtained.

The article "MUC1 gene silencing inhibits proliferation, invasion, and migration while promoting apoptosis of oral squamous cell carcinoma cells" was retracted in 2020. Reason: manipulated images.

### Immunohistochemical staining

The specimens were embedded in paraffin wax and sliced. The slices dehydrated with gradient ethanol, inactivated endogenous enzyme with H_2_O_2_ and rinsed with phosphate buffer saline (PBS) three times 5 min each time. The slices were incubated with normal goat serum at room temperature for 15 min, added with the primary antibody of 20–30 μl PBS diluted MUC1 (1:100, Abcam, Cambridge, U.K.) and Slug (1:100, Abcam, Cambridge, U.K.) for incubation at 4°C overnight. The PBS replaced the primary antibody as a negative control. After that, the slices were rinsed with PBS three times, incubated with biotin labeled secondary antibody for 20 min, incubated with horseradish enzyme labeled streptomyces ovalbumin working fluid for 20 min and developed with diaminobenzidine (DAB) for 3–5 min (Beijing Zhongshan Golden Bridge Biotechnology Co., Ltd., Beijing, China). Next, the slices were washed with running water, counterstained with hematoxylin for 5 min, dehydrated, cleared by xylene, and sealed. The PBS replaced the primary antibody as a blank control. Five high-power visual fields were randomly selected to observe the positive expression of MUC1 and Slug.

### Cell culture

Normal oral epithelial cell line HOK and OSCC cell line SCC-4, Cal-27, TSCCA, and Tca8113 were purchased from American Type Culture Collection. Normal oral epithelial cell line HOK was cultured in HOK cell culture medium (Scien Cell, U.S.A.), SCC-4 and Cal-27 OSCC cells were cultured in DMEM (with 100 U/ml penicillin and 100 μg/ml streptomycin) containing 10% FBS, and TSCCA and Tca8113 OSCC cells were cultured in RPMI-1460 medium (with 10% FBS, 100 U/ml penicillin and 100 μg/ml streptomycin). All the cells were cultured in an incubator with 5% CO_2_ and 95% relative humidity at 37°C. The cells in logarithmic growth phase were collected and subcultured every 2 days.

### Preparation of recombinant expression plasmid, cell transfection, and grouping

Two siRNA oligonucleotide sequence for MUC1 gene were designed: MUC1 siRNA-1 sequence: 5′-AAGGTACCATCAATGTCCACG-3′, MUC1 siRNA-2 sequence: 5′-AAGTTCAGTGCCCAGCTCTAC-3′. At the same time, a NC sequence (siRNA-NC) was designed: 5′-CGCTTACCGATTCAGAATGG-3′. Two siRNA recombinant expression plasmids pGC-LV-MUC1 siRNA-1 and pGC-LV-MUC1 siRNA-2 were constructed using lentiviral plasmid pGC-LV. The recombinant plasmid was successfully digested and sequenced to confirm the successful recombination. The siRNA sequence was synthesized by Shanghai Genechem Co., Ltd. (Shanghai, China). TSCCA cells were inoculated into a cell culture plate at a density of 1 × 10^9^ cells/l. The multiplicity of infection of viral plasmid was set as 50, and the cell transfection and grouping of TSCCA cells were based on transfection kit steps: (1) blank group: no virus infection; (2) con-siRNA group: infected with empty pGC-LV; (3) siRNA-NC group: infected with pGC-LV-siRNA-NC; and (4) MUC1 siRNA-2 group: infected with pGC-LV-MUC1 siRNA-2.

The article "MUC1 gene silencing inhibits proliferation, invasion, and migration while promoting apoptosis of oral squamous cell carcinoma cells" was retracted in 2020. Reason: manipulated images.

### MTT assay

When the transfected TSCCA cells reached about 80%, the cells were washed with PBS twice. The cells were detached by trypsin, and the single cell suspension was made by trituration through the straw. The inoculated cells were inoculated in a 96-well plate at density of 3 × 10^3^ – 6 × 10^3^ cells in each well (200 μl/well), and six parallel wells were set. After incubated in a CO_2_ incubator at 37°C for 24–72 h, MTT solution (5 mg/ml, Sigma–Aldrich, St. Louis, MO, U.S.A.) was added to each well. The MTT solution (250 mg) was put it in a beaker, added with 50 ml of PBS (0.01 mol/l, pH 7.4), and stirred for 30 min on an electromagnetic mixer in in normal environment. The microporous filtering film (0.22 μm) was used for degerming, packaged and reserved at 4°C for further use. Next, after incubating in a CO_2_ incubator at 37°C for 4 h, and the culture medium was abandoned. Each well was added with 150 μl DMSO, shaking gently for 10 min to dissolve crystal. The optical density (OD) value of every well was determined with a microplate reader at 0, 24, 48, and 72 h, respectively. The OD value was set as ordinate, and the interval time was set as horizontal ordinate to plot MTT curve. The experiment was repeated three times.

### EdU assay

The DNA replication of the cells was measured using a Cell-light EdU Luminescence Assay Kit (RiboBio, Guangzhou, China). Each group of cells was routinely detached, resuspended and counted, and seeded in a 96-well plate at 1.0 × 10^4^ cells/well, with three replicate wells in each group. After incubating for 2 h with 100 μl of 50 μM EdU, cells were rinsed with PBS and fixed with 4% paraformaldehyde for 30 min at room temperature. Next, the cells were rinsed with 0.5% Triton X-100, stained with 100 μl 1 × Apollo^®^ staining solution, and incubated for 30 min. Subsequently, the cells were rinsed with 0.5% Triton X-100, stained with 100 μl 1 × Hoechst 33342 staining solution, and incubated for 30 min. Pictures were taken under a fluorescence microscope to calculate the number of cells with EdU label (red) and unlabeled (blue). Labeling index = (number of labeled [red] cells/number of labeled [red] cells + number of unlabeled [blue] cells) × 100%.

The article "MUC1 gene silencing inhibits proliferation, invasion, and migration while promoting apoptosis of oral squamous cell carcinoma cells" was retracted in 2020. Reason: manipulated images.

### Colony formation assay

After 72 h of transfection, the cells in logarithmic growth phase were inoculated in a six-well culture plate (200 cells per well). Three parallel wells were set up and cultured at rest for 2 weeks. When white colony spots were observed in the naked eye, the operation was terminated. The cells were fixed with methanol (2 ml) at room temperature for 15 min, then stained with Giemsa solution at room temperature for 15 min, washed with water slowly, and dried. Cell colonies with more than 50 cells were counted under an optical microscope and the colony formation rate was calculated as the number of colonized cells/inoculated cells × 100%. The experiment was repeated three times.

### Flow cytometry

The cells were seeded into six-well culture plates according to 1 × 10^6^ cells per well. After cell adherence, cells were cultured synchronously for 12 h, then the original culture medium was discarded, and the corresponding treatment was given for a specific time. The cell culture medium was carefully collected into a sterile centrifuge tube, with the trypsin to detach the cells. When the cells could be gently pipetted with a pipette, the cells were added with the previously collected cell culture solution. All the adherent cells were triturated for scattering cells. The cell suspension was collected, and the cells were centrifuged to the bottom of the tube, with the supernatant discarded. After that, the cells were washed with PBS twice, resuspended with precooled 75% ethanol, and fixed overnight at −20°C. After centrifugation, the supernatant was removed, and the cells were rinsed with PBS twice. The cells were collected by centrifugation, and 500 μl of PBS (containing 50 mg/ml propidium iodide [PI] and 50 μg/ml RNAse A) was added to each sample, then mixed together, and placed in water-bath at 37°C for 30 min. After centrifugation, the supernatant was abandoned, and the cells were suspended with PBS. Cell cycle distribution was measured and analyzed by flow cytometer (BD FACSAria™, BD Biosciences, San Jose, CA, U.S.A.). The experiment was repeated three times independently.

After 72 h of transfection, the cells were collected, rinsed with PBS three times, and then added to the precooled 1 × binding buffer (500 μl). Next, the cell suspensions were added with 5 μl Annexin-V-FITC and 2.5 μl PI and mixed gently. The cell apoptosis was detected by flow cytometer (BD FACSAria™, BD Biosciences, San Jose, CA, U.S.A.). In the scattered plot, the lower left quadrant (Q4) showed healthy living cells (FITC^−^/PI^−^), the lower right quadrant (Q3) showed early apoptotic cells (FITC^+^/PI^−^), the right upper quadrant (Q2) showed necrosis and late apoptosis cells (FITC^+^/PI^+^), and apoptosis rate = early apoptosis percentage (Q3) + late apoptosis percentage (Q2). The experiment was repeated three times independently.

The article "MUC1 gene silencing inhibits proliferation, invasion, and migration while promoting apoptosis of oral squamous cell carcinoma cells" was retracted in 2020. Reason: manipulated images.

### Scratch test

The back of the six-well plate was perpendicular to the horizontal axis and marked with a marker at every 0.5–1.0 cm interval. Cells were inoculated in each well. When the cells grew to 90% confluence, the cells were treated with mitomycin C (10 μg/ml, Sigma, St. Louis, MO, U.S.A.) for 2 h, and washed with PBS three times. The cells were scratched along the marking line using a gun head perpendicular to the plate and washed twice with PBS to remove the floating cells. The cells were supplemented with serum-free medium and placed under the conditions of saturated humidity with 5% CO_2_ at 37°C. Photographs were taken under an inverted microscope at 0 and 24 h. Image tool software (Bechtel Nevada, Los Alamos Operations) was used to calculate healing area, and the healing rate was: (width value of initial scratch − width value of current scratch)/width value of initial scratch × 100%. The experiment was repeated three times.

### Transwell assay

Preparation of single cell suspension from serum-free medium was conducted by conventional method, with 5 × 10^5^ cells/ml. Matrigel was dissolved overnight at 4°C. The Matrigel was diluted with serum-free medium at the ratio of 1:3, and 30 μl diluted Matrigel was added into the apical chamber in each Tanswell chamber in three times (15, 7.5, and 7.5 μl) (Corning, New York, U.S.A.). At intervals of 10 min, the Matrigel was evenly spread and all micropores on the bottom of the apical chamber were covered. The medium containing 10% FBS was added to the basolateral chamber of 24-well plate with the cells suspensions inoculated into the apical chamber of Transwell and incubated at 37°C for 24 h. After removing the chamber and aspirating the medium, the cells that had not passed through the membrane were gently wiped off with a cotton swab and fixed it with 4% paraformaldehyde for 30 min. After natural air drying, the cells were stained with crystal violet for 5 min, washed gently with distilled water several times and air-dried. The number of cells passing through the Matrigel was used as an indicator of invasion. The experiment was repeated three times.

The article "MUC1 gene silencing inhibits proliferation, invasion, and migration while promoting apoptosis of oral squamous cell carcinoma cells" was retracted in 2020. Reason: manipulated images.

### Reverse transcription quantitative PCR

TRIzol method (Takara, Dalian, China) was used to extract total RNA in cells and tissues to determine the concentration and purity of RNA. The sample RNA was reversed to cDNA according to the specifications of the Reverse Transcription Kit (DRR047S, Takara Biomedical Technology [Dalian] Co., Ltd), and the total system was 10 μl. The cDNA obtained from the above inversion was added with 65 μl diethyl pyrocarbonate water to dilute and mix well. The primers were synthesized by Shenzhen BGI Co., Ltd. (Shenzhen, China). MUC1-Forward: 5′-TCAGTGCCGCCGAAAGAAC-3′, MUC1-Reverse: 5′-GCTCATAGGATGGTAGGTATCCC-3′; glyceraldehyde phosphate dehydrogenase (GAPDH)-Forward: 5′-AACGGATTTGGTCGTATTGGG-3′, GAPDH-Reverse: 5′-TCGCTCCTGGAAGATGGTGAT-3′. GAPDH was an internal reference, with three repeats for per gene in each sample. The reliability of PCR results was evaluated by the dissolution curve. ΔCT = CT_(target gene)_ − CT_(internal reference)_, ΔCT = ΔCT_(experimental group)_ − ΔCT_(control group)_. The relative expression of target gene was calculated by 2^−ΔΔ*C*^_T_ [25]. The experiment was repeated three times.

### Western blot analysis

The total protein was extracted from the tissues and cells of each group. The bicinchoninic acid protein concentration assay kit was used to measure protein concentration, and the protein concentration of each group was adjusted. After adding with 5 × SDS loading buffer, the cells were denatured at 95°C for 5 min, separated by SDS PAGE, transferred, added with 5% skim milk powder, and sealed overnight at 4°C. After the membrane was washed with Tris-buffered saline with Tween-20 (TBST), it was then added with the primary antibody MUC1 (1:1000, Abcam, Cambridge, U.K.), Slug (1 μg/ml, Abcam, Cambridge, U.K.), E-cadherin (1:50, Abcam, Cambridge, U.K.), Vimentin (1:500, Abcam, Cambridge, U.K.) and GAPDH (1:1000, Millipore Inc., Billerica, MA, U.S.A.), and incubated overnight at 4°C. After the membrane was washed with TBST, it was then added with horseradish peroxidase-labeled secondary antibody and incubated overnight at 4°C. After the membrane was washed with TBST, enhanced chemiluminescence was used for developing. The gray value of the target band was analyzed by ImageJ software, and the experiment was repeated three times independently.

### Statistical analysis

SPSS 19.0 (IBM-SPSS Inc, Chicago, IL, U.S.A.) software was used for data analyzing, and the experiment was repeated three times independently to calculate mean and standard deviation. The t test was used to analyze the difference between groups. One-way ANOVA was used to analyze the difference amongst multigroups. After ANOVA, pairwise comparisons were analyzed by the least significant difference t test (LSD-t). The enumeration data were expressed by rate or percentage, which was analyzed by χ^2^ test. Bilateral analysis was used in all analyses, and significant differences were observed in *P*<0.05.

The article "MUC1 gene silencing inhibits proliferation, invasion, and migration while promoting apoptosis of oral squamous cell carcinoma cells" was retracted in 2020. Reason: manipulated images.

## Results

### Higher positive rate of MUC1 and Slug expression in OSCC tissue

With the aim to observe the expression of MUC1 in OSCC tissues and normal oral mucosa tissues, we performed immunohistochemistry to detect the expression of MUC1. To further investigate whether MUC1 acts on OSCC via Slug, we used immunohistochemistry to detect the expression of Slug. The immunohistochemical staining results demonstrated that MUC1 was mainly expressed in cell cytoplasm in light yellow to brown in OSCC and normal oral mucosa tissues, and the nucleus was basically not stained (Figure 1). The positive rate of MUC1 in OSCC tissues was 66.67% (60/90), which was significant different that in the normal oral mucosa tissues (17.14%; 6/35; Table 1). The positive rate of Slug in OSCC tissues was 73.33% (66/90), which was higher than that in normal oral mucosa tissues (14.28%; 5/35; Table 1). According to Spearman correlation analysis, MUC1 expression was positively correlated with Slug expression (r = 0.731, *P*<0.001). To analyze the correlation between the expression of MUC1 and the clinicopathological features of OSCC tissues, the results showed that the positive rate of MUC1 expression in OSCC tissues was associated with differentiation degree and lymph node metastasis (both *P*<0.05). The positive expression rate of MUC1 increased with the degree of tumor differentiation. The positive expression rate of MUC1 in patients without lymph node metastasis was significantly lower than that in patients with lymph node metastasis. However, the expression of MUC1 was not related to gender and age of patients (both *P*>0. 05; Table 2).

**Figure 1:** Higher expression of MUC1 and Slug are found in OSCC tissues by immunohistochemical staining; **OSCC tissues = 90 and normal oral mucosa tissues** = 35

**Table 1:** Expression of MUC1 and Slug in the OSCC group and the control group

	OSCC	Control	*P*
MUC1			<0.001
Positive (n)	60	6	
Negative (n)	30	29	
Positive expression rate (%)	66.67	17.14	
Slug			<0.001
Positive (n)	66	5	
Negative (n)	24	30	
Positive expression rate (%)	73.33	14.28	

The enumeration data were expressed by rate or percentage, which was analyzed by χ^2^ test.

**Table 2:** Relationship between expression of MUC1 protein and clinicopathological parameters in OSCC

Clinical features	Case	MUC1 expression		*P*
		(+)	(-)	
Gender				0.121
Male	46	27 (45.00%)	19 (63.33%)	
Female	44	33 (55.00%)	11 (36.67%)	
Age (years)				0.878
<60	35	23 (38.33%)	12 (40.00%)	
≥60	55	37 (61.67)	18 (60.00%)	
Differentiation degree				0.003
High	30	13 (21.67%)	17 (56.67%)	
Moderate	30	22 (36.67%)	8 (26.67%)	
Low	30	25 (41.66%)	5 (16.66%)	
Lymph node metastasis				0.028
Yes	42	33 (55.00%)	9 (30.00%)	
No	48	27 (45.00%)	21 (70.00%)	

The data were expressed in rate or percentage, and the analysis was conducted by χ^2^ test.

The article "MUC1 gene silencing inhibits proliferation, invasion, and migration while promoting apoptosis of oral squamous cell carcinoma cells" was retracted in 2020. Reason: manipulated images.

### Higher expression of MUC1 mRNA and protein is found in OSCC cells

Subsequently, in order to observe the expression of MUC1 in OSCC tissues and normal oral mucosa tissues, we adopted RT-qPCR and western blot analysis to detect the expression of mRNA and protein of MUC1 in tissue samples. The results suggested that the expression of MUC1 mRNA and protein in OSCC tissues was higher than that in normal oral mucosa tissues (*P*<0.05; Figure 2A). Additionally, mRNA and protein expression of MUC1 in normal oral epithelial cell line HOK and OSCC cell line SCC-4, Cal-27, TSCCA, and Tca8113 were detected by RT-qPCR and western blot analysis. The results suggested that the expression of MUC1 mRNA and protein in OSCC cell line SCC-4, Cal-27, TSCCA, and Tca8113 was higher than that in normal oral epithelial cell line HOK (*P<*0.05; Figure 2B). The expression of MUC1 was the highest in TSCCA cells, so we have chosen it for subsequent interference test.

**Figure 2:** Higher expression of MUC1 mRNA and protein is found in OSCC tissues and cells (**A**) Expression of MUC1 mRNA and protein in OSCC tissues and normal oral mucosa tissues, OSCC tissues = 90, normal oral mucosa tissues = 35; (**B**) mRNA and protein expression of MUC1 in normal oral epithelial cell line HOK and OSCC cell line SCC-4, Cal-27, TSCCA, and Tca8113. *P<0.05 vs normal oral epithelial cell line HOK. Data analysis was performed by *t*-test or one-way ANOVA. After one-way ANOVA, the LSD-t test was utilized for pairwise comparison.

### Expression of MUC1 in each group after transfection

Next, for the purpose of observing the effect of MUC1 silencing on MUC1 expression in OSCC cells, we used RT-qPCR and western blot analysis to detect the expression of MUC1 mRNA and protein in each group. First, we extracted the total RNA from the cells after 48 h of lentivirus infection of TSCCA cells, and RT-qPCR was then used to detect the expression of MUC1 in each group. The results (Figure 3A) indicated that compared with the blank group (uninfected TSCCA cells), the mRNA expression of MUC1 was significantly decreased in the MUC1 siRNA-1 group (1.00 ± 0.02 vs 0.37 ± 0.03, *P*<0.05) and the MUC1 siRNA-2 group (1.00 ± 0.02 vs 0.25 ± 0.02, *P*<0.05). Amongst them, the MUC1 mRNA expression in the MUC1 siRNA-2 group was significantly decreased, and the subsequent experiments were performed using MUC1 siRNA-2. There was no significant difference in MUC1 mRNA expression between the con-siRNA group (transfected with empty pGC-LV) and the siRNA NC group (transfected with pGC-LV-siRNA-NC) in comparison to the blank group (1.02 ± 0.06 vs 1.00 ± 0.02, *P*>0.05; 0.97 ± 0.08 vs 1.00 ± 0.02, *P>*0.05). The total protein was extracted by TSCCA cells infected with lentivirus for 72 h. The expression of MUC1 protein was detected by western blot analysis, and the results (Figure 3B) indicated that compared with the blank group, the protein expression of MUC1 was significantly decreased in the MUC1 siRNA-1 group and the MUC1 siRNA-2 group (0.76 ± 0.06 vs 0.29 ± 0.03, *P*<0.05; 0.76 ± 0.06 vs 0.15 ± 0.03, *P>*0.05). The protein expression of MUC1 was significantly decreased in the MUC1 siRNA-2 group, and the subsequent experiments were interfered with MUC1 siRNA-2. There was no significant difference in MUC1 protein expression amongst the con-siRNA group, the siRNA NC group and the blank group (0.74 ± 0.08 vs 0.76 ± 0.06, *P>*0.05; 0.78 ± 0.08 vs 0.76 ± 0.06, *P>*0.05).

The article "MUC1 gene silencing inhibits proliferation, invasion, and migration while promoting apoptosis of oral squamous cell carcinoma cells" was retracted in 2020. Reason: manipulated images.

**Figure 3:** MUC1 gene silencing suppresses proliferation of OSCC cells (**A**) Expression of MUC1 mRNA in TSCCA cells of each group after 48-h infection of empty lentiviral vector, recombinant lentivirus that interferes with MUC1 expression, and negative control; (**B**) expression of MUC1 protein in TSCCA cells of each group after 72-h infection of empty lentiviral vector, recombinant lentivirus that interferes with MUC1 expression, and negative control; (**C**) cell proliferation curve of cells in each group; (**D**) EdU assay for detection of DNA replication of cells; (**E**) cell colony formation rate in each group. Blank group: no virus infection; con-siRNA group: infected with empty pGC-LV; siRNA-NC group: infected with pGC-LV-siRNA-NC; MUC1 siRNA-2 group: infected with pGC-LV-MUC1 siRNA-2. *P<0.05 vs the blank group. Data analysis was performed by one-way ANOVA. After one-way ANOVA, the LSD-t test was utilized for pairwise comparison. The experiment was repeated three times.

### Silencing of MUC1 inhibits the proliferation of OSCC cells

In order to observe the effect of interfering MUC1 expression on the proliferation of OSCC cells, we performed the MTT assay. As shown in Figure 3C, at 0 and 24 h after transfection, the OD_450nm_ value of the blank group, con-siRNA group, siRNA NC group, and MUC1 siRNA-2 group were 0.38 ± 0.03 vs 0.37 ± 0.04 vs 0.37 ± 0.03 vs 0.38 ± 0.04 and 0.60 ± 0.04 vs 0.55 ± 0.06 vs 0.57 ± 0.04 vs 0.50 ± 0.05, respectively (*P>*0.05). At 48 and 72 h after transfection, the OD_450nm_ value of the blank group, con-siRNA group, siRNA NC group, and MUC1 siRNA-2 group were 0.94 ± 0.06 vs 0.89 ± 0.07 vs 0.91 ± 0.06 vs 0.64 ± 0.05 and 1.26 ± 0.08 vs 1.20 ± 0.08 vs 1.22 ± 0.07 vs 0.80 ± 0.07, respectively. The OD_450nm_ value in the MUC1 siRNA-2 group was lower than that in the blank group, con-siRNA group and siRNA NC group (*P<*0.05). No significant difference was found amongst the blank group, con-siRNA group and siRNA NC group (*P>*0.05).

The article "MUC1 gene silencing inhibits proliferation, invasion, and migration while promoting apoptosis of oral squamous cell carcinoma cells" was retracted in 2020. Reason: manipulated images.

EdU is a thymidine analog with an acetylenic group attached to it that is rare in natural compounds. It replaces thymine (T) in the DNA replication phase and penetrates into the DNA molecule being synthesized. Based on Apollo^®^-based fluorescence, the specific reaction of the dye with EdU allows direct and accurate detection of DNA replication. The DNA replication of cells was detected by EdU assay. The results suggested that the proportion of EdU-positive cells in the blank, con-siRNA, siRNA NC, and MUC1 siRNA-2 groups was 46.5 ± 2.5%, 45.0 ± 1.6%, 44.5 ± 2.2%, and 30.4 ± 2.0%, respectively. No significant difference was found amongst the blank, con-siRNA group and siRNA NC groups (*P>*0.05). When TSCCA cells interfered with MUC1, the DNA replication of the cells was significantly decreased (*P<*0.05) (Figure 3D).

In order to observe the effect of interfering MUC1 expression on the colony formation of OSCC cells, we performed the colony formation assay. As shown in Figure 3E, the colony formation rate in the MUC1 siRNA-2 group was 21.45% ± 2.02%, which was significantly lower than that of the blank group (54.81 ± 5.89%), con-siRNA group (52.02 ± 5.63%), and the siRNA NC group (53.01 ± 5.62%) (*P<*0.05). There was no significant difference in colony formation rate amongst the blank group, con-siRNA group, and the siRNA NC group (*P>*0.05). These results suggest that interference with MUC1 gene can inhibit the proliferation of OSCC cells.

### MUC1 gene silencing inhibits cell cycle progression and induces apoptosis of OSCC cells

Flow cytometry was used to detect the effects of interfering with MUC1 on cell cycle and apoptosis of OSCC cells. The cell cycle results showed that (Figure 4A) in the blank group, the cells in G1 phase were 54.86 ± 3.21%, in G2 phase was 16.45 ± 1.25%, and in S phase was 27.69 ± 2.04%; in the con-siRNA group, the cells in G1 phase were 54.36 ± 3.78%, in G2 phase was 17.64 ± 1.22%, and in S phase was 28.00 ± 1.99%; the cells in G1 phase in the siRNA NC group were 54.42 ± 3.68%, in G2 phase, 17.32 ± 1.24%, and in S phase, 28.26 ± 1.94%; in the MUC1 siRNA-2 group, the cells in G1 phase were 70.88 ± 3.58%, in G2 phase, 8.76 ± 0.72% and in S phase, 20.36 ± 1.63%. In contrast with the blank group, the cells in G1 phase increased and those in G2 phase decreased in the MUC1 siRNA-2 group (*P<*0.05). There was no significant difference in cell cycle distribution amongst the blank group, con-siRNA group, and the siRNA NC group (*P>*0. 05).

The article "MUC1 gene silencing inhibits proliferation, invasion, and migration while promoting apoptosis of oral squamous cell carcinoma cells" was retracted in 2020. Reason: manipulated images.

**Figure 4:** MUC1 gene silencing represses cell cycle entry and induces apoptosis of OSCC cells (**A**) Comparison of cell cycle distribution in each group; (**B**) comparison of cell apoptosis in different groups. Blank group: no virus infection; con-siRNA group: infected with empty pGC-LV; siRNA-NC group: infected with pGC-LV-siRNA-NC; MUC1 siRNA-2 group: infected with pGC-LV-MUC1 siRNA-2. *P<0.05 vs the blank group. Data analysis was performed by one-way ANOVA. After one-way ANOVA, the LSD-t test was utilized for pairwise comparison. The experiment was repeated three times.

The results of cell apoptosis showed that (Figure 4B) the cell apoptosis rate in the blank, con-siRNA, siRNA NC, and MUC1 siRNA-2 groups was 4.9 ± 0.7%, 4.7 ± 0.6%, 4.8 ± 0.6%, and 14.8 ± 0.9%, respectively. The cell apoptosis rate in the blank, con-siRNA and siRNA NC groups was lower than that in the MUC1 siRNA-2 groups (*P<*0.05). There was no significant difference in cell cycle distribution amongst the blank group, con-siRNA group and the siRNA NC group (*P>*0.05). These results suggest that silencing of MUC1 gene induces apoptosis of OSCC cells.

### MUC1 gene silencing decrease Slug expression and inhibits the development of EMT in OSCC cells

We detected the expression of Slug, E-cadherin, and Vimentin by western blot analysis to observe the MUC1 gene silencing on expression of Slug, epithelial interstitial marker proteins E-cadherin, and Vimentin of OSCC cells (Figure 5A,B). In contrast with the blank group, the expression of E-cadherin was increased and expression of Slug and Vimentin was decreased in the MUC1 siRNA-2 group (E-cadherin: 0.08 ± 0.02 vs 0.17 ± 0.03; Slug: 0.45 ± 0.05 vs 0.21 ± 0.05; Vimentin: 0.24 ± 0.04 vs 0.11 ± 0.03, *P<*0.05). The expression of Slug, E-cadherin, and Vimentin was not significantly differed amongst the blank, con-siRNA and the siRNA-NC groups (0.45 ± 0.05 vs 0.43 ± 0.06 vs 0.44 ± 0.07; 0.08 ± 0.02 vs 0.09 ± 0.03 vs 0.08 ± 0.03; 0.24 ± 0.04 vs 0.23 ± 0.04 vs 0.22 ± 0.03, *P<*0.05). These results suggest that MUC1 gene silencing can decrease Slug expression and prevent the occurrence of EMT in OSCC cells.

**Figure 5:** MUC1 gene silencing decreases expression of Slug and inhibits the development of EMT in OSCC cells (**A**) Protein bands of Slug, E-cadherin, and Vimentin in each group; (**B**) expression of Slug, E-cadherin, and Vimentin in each group. Blank group: no virus infection; con-siRNA group: infected with empty pGC-LV; siRNA-NC group: infected with pGC-LV-siRNA-NC; MUC1 siRNA-2 group: infected with pGC-LV-MUC1 siRNA-2. *P<0.05 vs the blank group. Data analysis was performed by one-way ANOVA. After one-way ANOVA, the LSD-t test was utilized for pairwise comparison. The experiment was repeated three times.

The article "MUC1 gene silencing inhibits proliferation, invasion, and migration while promoting apoptosis of oral squamous cell carcinoma cells" was retracted in 2020. Reason: manipulated images.

### MUC1 gene silencing inhibits migration and invasion in OSCC cells

Transwell assay was used to detect the invasion ability of each group, and scratch test was used to detect the migration ability of each group. The results of Transwell assay (Figure 6A) showed that compared with the blank group, the number of cells invading the membrane decreased significantly in the MUC1 siRNA-2 group (88 ± 4 vs 48 ± 6, *P<*0.05). There was no significant difference in cell invasion amongst the blank group, con-siRNA group and the siRNA NC group (88 ± 4 vs 85 ± 7, *P>*0. 05; 88 ± 4 vs 86 ± 6, *P>*0.05). The scratch test results revealed that (Figure 6B) compared with the blank group, the scratch repair rate decreased significantly in the MUC1 siRNA-2 group (51.23 ± 4.95% vs 30.26 ± 3.68%, *P<*0.05). There was no significant difference amongst the blank group, con-siRNA group and the siRNA NC group (51.23 ± 4.95% vs 48.86 ± 5.21%, *P>*0.05; 51.23 ± 4.95% vs 49.97 ± 5.03%, *P>*0.05). These results suggest that silencing of MUC1 gene can prevent the invasion and migration in OSCC cells.

**Figure 6:** MUC1 gene silencing inhibits migration and invasion in OSCC cells (**A**) Invasive ability of cells in each group; (**B**) migration ability of cells in each group. Blank group: no virus infection; con-siRNA group: infected with empty pGC-LV; siRNA-NC group: infected with pGC-LV-siRNA-NC; MUC1 siRNA-2 group: infected with pGC-LV-MUC1 siRNA-2. *P<0.05 vs the blank group. Data analysis was performed by one-way ANOVA. After one-way ANOVA, the LSD-t test was utilized for pairwise comparison. The experiment was repeated three times.

## Discussion

OSCC is the most common neoplasm in the oral cavity, which has poor clinical outcomes related to recurrence and metastasis [26,27]. Despite of the recent progress has been made in the diagnosis of together with the therapeutic modalities for OSCC, the 5-year OS rate has not been improved [28]. Thus, early prevention, detection as well as treatment would be the key point for the improvement of the survival rate and quality of life of patients suffering from OSCC patients [29,30]. Therefore, it is urgently needed to seek for new targets for the effective therapy through a more comprehensive understanding of the mechanism of OSCC. Collectively, MUC1 gene silencing can inhibit the proliferation, invasion, and migration while inducing apoptosis of OSCC cells.

The article "MUC1 gene silencing inhibits proliferation, invasion, and migration while promoting apoptosis of oral squamous cell carcinoma cells" was retracted in 2020. Reason: manipulated images.

First, our study showed that higher expression of MUC1 was found in OSCC tissues and cells. As previously reported, MUC1 is frequently up-regulated in various cancers, which is also regarded as a potential biomarker for diagnosis, prognosis, and therapy of cancers [31]. Many researches have demonstrated that MUC1, as an oncogenic protein, is overexpressed in ovarian, gastric cancer as well as acute myeloid leukemia [32,33]. Additionally, MUC1 has been suggested to be up-regulated in a great many of cancer types, such as breast cancer, gastric cancer as well as type B3 thymoma and thymic carcinoma [34–36]. Furthermore, a previous study revealed that both transcription and translation products of MUC1 presented high expression in OSCC-derived cell lines [37]. All these mentioned above confirmed the results of our study.

Meanwhile, the findings of our study also suggested that silencing of MUC1 inhibited the proliferation, cell cycle progression and EMT while inducing apoptosis of OSCC cells. The involvement of mucins has also been proposed in the renewal and differentiation of the epithelium, and also, in the modulation of both cell adhesion and cell signaling [38]. Similar to our study, a previous study has found that silencing of MUC1 is able to inhibit cell proliferation though the activation of apoptosis pathways and the induction of apoptosis in PANC-1 cells [39]. Additionally, another study has indicated that silencing of MUC1 is capable of inhibiting the development of non-small cell lung cancer cells [17]. As for the role of MUC1 in OSCC, it could be explained by the following reasons. Studies have also demonstrated that MUC1 enables to interact with several signals that involving in cell adhesion, growth as well as survival, and these signals includes protein kinase C, c-Src, and family member of the human epidermal growth factor receptor [18,40]. In addition, MUC1 is closely related to other molecules, including β-catenin, or epidermal growth factor receptor, which is able to regulate transcription of different genes that is responsible for progression and invasiveness of cancer [41]. Besides, MUC1 results in the initiation of several signaling pathways, which could promote growth, migration, invasion, as well as metastasis of tumors [42]. Furthermore, MUC1 enhances invasion and metastasis, and promotes EMT via up-regulating the expressions of transcription factors, such as Snail and Slug, as well as down-regulation of E-cadherin expression [23]. It is reported that Slug has an essential role in the regulation of EMT by inhibiting several epithelial markers together with adhesion molecules, including E-cadherin [43]. E-cadherin is known as an important factor for EMT, and the loss of E-cadherin has been discussed in invasion and metastasis of many cancers [44]. Slug (Snail2) is an EMT transcription factor with zinc finger structure. Various signaling molecules and transduction pathways are involved in the regulation of Slug expression. The zinc finger transcription factor Slug mainly participates in EMT by regulating E-cadherin [45]. Slug is an invasion-promoting factor that inhibits E-cadherin transcription and enhances tumor cell migration and invasion [22]. These results suggest that Slug plays an important role in cell invasion and migration. It is reported that the activation of Slug results in a reduction in the proliferation of human epidermal keratinocytes [46], and ectopic expression of Slug in the developing neural tube results in reduced cell proliferation [47], suggesting that Slug has a close association with cell proliferation. In addition, evidence has shown that Slug promotes survival and hinders cell death by directly repressing PUMA, a key BH3-only antagonist of the antiapoptotic Bcl-2 protein [48]. Bcl-2 is a Slug-regulated gene in mouse [49]. siRNA directed against the Slug gene increases cell death induction in human melanoma cell lines exposed to cisplatin and fotemustine [50], suggesting Slug has a close association with cell apoptosis. Based on the above findings, we hypothesized that MUC1 may affect cell proliferation, apoptosis, invasion, migration, and EMT through the action of Slug. The results in our study showed that the positive expression rate of Slug protein in OSCC group was higher than that in the control group; the expression of MUC1 was positively correlated with Slug expression; MUC1 gene silencing can reduce the expression of Slug. In summary, MUC1 gene silencing can inhibit proliferation, invasion, migration, EMT while promoting apoptosis of OSCC cells via the inhibition of Slug.

The article "MUC1 gene silencing inhibits proliferation, invasion, and migration while promoting apoptosis of oral squamous cell carcinoma cells" was retracted in 2020. Reason: manipulated images.

In conclusion, our study highlights the function of MUC1 in OSCC. Additionally, MUC1 gene silencing can inhibit the proliferation, invasion, and migration while inducing apoptosis of OSCC cells. However, the potential mechanisms of MUC1 in the progression of OSCC needs further explanation. Meanwhile, we would carry out immunohistochemical serial section to detect the MUC1 and Slug protein expression to further verify our results.

## Abbreviations

DAB: diaminobenzidine
EMT: epithelial-mesenchymal transition
LSD-t: least significant difference t test
MUC1: mucin 1
OD: optical density
OSCC: oral squamous cell carcinoma
PBS: phosphate buffer saline
PI: propidium iodide
TBST: Tris-buffered saline with Tween-20
WHO: World Health Organization
